The article "Polydatin protects H9c2 cells from hypoxia-induced injury via up-regulating long non-coding RNA DGCR5" was retracted in 2020. Reason: concerns about the data.

# Polydatin protects H9c2 cells from hypoxia-induced injury via up-regulating long non-coding RNA DGCR5

**DOI:** 10.1590/1414-431X20198834

**Published:** 2019-12-05

**Authors:** Jinhua Dai, Jianbo Ma, Yufeng Liao, Xianhai Luo, Guofang Chen

**Affiliations:** 1 Department of Clinical Laboratory, Hwa Mei Hospital, University of Chinese Academy of Sciences (Ningbo No. 2 Hospital), Ningbo, Zhejiang, China; 2 Department of Clinical Laboratory, Ningbo Kangning Hospital, Ningbo Mental Health Center, Ningbo, Zhejiang, China; 3 Department of Cardiology, Hwa Mei Hospital, University of Chinese Academy of Sciences (Ningbo No. 2 Hospital), Ningbo, Zhejiang, China

**Keywords:** Myocardial infarction, Apoptosis, Autophagy, PI3K/AKT/mTOR pathway, MEK/ERK pathway

## Abstract

Polydatin (PD), a monocrystalline polyphenolic drug mainly found in the roots of *Polygonum cuspidatum*, has various pharmacological activities. Long non-coding RNAs (lncRNA) DiGeorge syndrome critical region gene 5 (DGCR5) was found to participate in the suppression of multiple cancers. Here, we proposed to study the effect of PD on myocardial infarction (MI) by inducing DGCR5. CCK-8 assay was performed to detect the viability of H9c2 cells. Flow cytometry was utilized to test apoptosis of H9c2 cells. These results determined the optimal concentration and effect time of hypoxia as well as PD. Si-DGCR5 was transfected into cells and the expression level was determined by qRT-PCR. Western blot was utilized to evaluate the expression of apoptosis-related proteins, Bcl-2, Bax, and cleaved-caspase-3, as well as autophagy-associated proteins including Beclin-1, p62, and LC3-II/LC3-I. As a result, PD efficiently attenuated hypoxia-induced apoptosis and autophagy in H9c2 cells. The expression of DGCR5 was down-regulated by hypoxia and up-regulated by PD. Besides, knocking-down the expression of DGCR5 inhibited the protection of PD in H9c2 cells. In addition, PD up-regulated the accumulation of DGCR5, DGCR5 decreased the expression of Bcl-2 and p62, raised the expression of Bax and cleaved-caspase-3, and the proportion of LC3-II/LC3-I. PD stimulated the PI3K/AKT/mTOR and MEK/ERK signaling pathways via up-regulating the expression of DGCR5. Our data demonstrated that PD reduced cell apoptosis and autophagy induced by hypoxia in cardiomyocytes. Moreover, PD activated PI3K/AKT/mTOR and MEK/ERK signaling pathways by up-regulating the expression of DGCR5.

## Introduction

Myocardial infarction (MI) is a prevalent clinical manifestation for ischemic heart disease and coronary artery disease (1). Generally, 3–4 million people have an MI annually (2). The manifestations of MI are varying degrees of chest pain, which can move to the left arm or left side of the neck, dyspnea, sweating, nausea, irregular heartbeat, apprehension, fatigue, etc. (3). The current treatment of MI is taking drugs that act to lower blood cholesterol and platelet aggregation, such as aspirin and tissue plasminogen activator (tPA). Besides that, several painkillers are recommended to relieve the pain associated with MI, such as morphine and meperidine (4). Although there is a wide variety of drugs used for MI, the mortality and morbidity of MI are still increasing. Currently, one million deaths are caused by MI annually (5). Thus, comprehensive research on prevention and treatment of MI is still necessary.

Polydatin (PD) is a monocrystalline polyphenolic pharmaceutical mainly found in the roots of *Polygonum cuspidatum* (6). Recent studies already have found that PD possesses numerous pharmacological functions including anti-cardiovascular, anti-inflammatory, and anti-oxidative effects (7). Zhang et al. (8) reported that PD alleviates myocardial dysfunction, augments autophagy, and improves mitochondrial bioenergy. Additionally, PD protects against acute MI-induced cardiac damage according to Chen et al. (9). Accumulating evidence indicates that PD plays a vital role in cardiac functions and other diseases. Notwithstanding all the research, the effects and potential molecular mechanisms of PD against MI are not well understood.

Long non-coding RNAs (lncRNAs) are a type of non-coding RNAs with a length ranging from 200 nucleotides to multiple kilobases (10). lncRNAs have no protein-coding ability and account for a large proportion of genomic transcripts (11). A vast amount of research determined that lncRNAs played vital roles in the regulation of several biological processes, including proliferation, DNA damage, differentiation, microRNA silencing, apoptosis, tumorigenesis, and metastasis (12,13). Many lncRNAs have been found to play a crucial role in MI. Huang et al. (14) reported that inhibition of lncRNA TTTY15 relieved hypoxia-induced myocardial cell injury by targeting miR-455-5p. The lncRNAs DiGeorge syndrome critical region gene 5 (DGCR5), also identified as Linc00037, was found to participate in the suppression of multiple cancers, such as papillary thyroid carcinoma, human laryngeal carcinoma, and gastric cancer (11,15,16). Previous research reported that under the treatment of hypoxia, DGCR5 suppressed neuronal apoptosis to improve acute spinal cord injury (17). As far as we know, the functional roles of DGCR5 in hypoxia injury to cardiomyocytes are rarely investigated.

Previous studies have demonstrated that PD protects against MI *in vivo* and *in vitro* (9). In the current research, we aimed to explore the effects of PD on hypoxia-induced MI. The underlying mechanism of DGCR5 was also studied. The findings of this study provided a novel insight for preventing MI.

## Material and Methods

### Cell culture

H9c2 cells (ATCC, USA) were derived from rat embryonic ventricular cardiomyocytes and incubated in Dulbecco's modified Eagle medium (DMEM, GIBCO, USA) containing 10% fatal bovine serum (FBS, GIBCO), 100 U/mL penicillin (Solarbio, China), and 100 µg/mL streptomycin (Wuhan Fortuna Chemical Co., Ltd., China) in an incubator that contained 95% air and 5% CO_2_ at 37°C.

### Cell treatment

PD was purchased from Meilun Biological Company (China) and diluted in dimethyl sulfoxide (DMSO). H9c2 cells were treated with PD for 24 h at the concentrations of 1, 3, 10, 15, and 20 μM. After incubation, the H9c2 cells were cultured in a hypoxia chamber, saturated with 94% N_2_, 5% CO_2_, and 1% O_2_ to reach a hypoxic status. Control cells were incubated in the normoxia conditions at 37°C in a humidified atmosphere of 95% air and 5% CO_2_.

### CCK-8 assay

Cell viability was determined with Cell Counting Kit-8 (CCK-8, Dojindo Laboratories, Japan). H9c2 cells were inoculated in a 96-well plate at a density of 5×10^3^ cells/well. When treatments were completed, the cell culture medium was substituted with fresh cell culture media containing 10 μL CCK-8, and then the cultures were incubated for 1 h at 37°C. Absorbance at 450 nm was determined using a microplate reader (Bio-Rad, USA).

### Determination of apoptosis

H9c2 cells were inoculated in a 6-well plate. After cells had been subjected to treatments as described above, cells were rinsed gently twice with cold phosphate buffered saline (PBS, Thermo Scientific, USA) and re-suspended in binding buffer. The rates of H9c2 cells apoptosis were analyzed by flow cytometry (Beckman Coulter, USA) following Annexin V-FITC/PI apoptosis detection kit (Beijing Biosea Biotechnology, China) instructions.

### Transfection

Si-negative control (NC) and si-DGCR5 were synthesized by and purchased from Shanghai GenePharma Co., Ltd. (China). All transfections were completed using Lipofectamine 3000 reagent (Invitrogen, USA) following the manufacturer's protocol. After H9c2 cells were transfected for 48 h, all cells were harvested for follow-up investigations.

### Real-time quantitative PCR

Total RNA was isolated from transfected H9c2 cells using Trizol reagent (Invitrogen), according to the manufacturer's instructions. RNA concentration and purity were measured by UV spectrophotometry (Multiskan FC Microplate Photometer, Thermo Scientific, Inc., USA) at 260 nm and 280 nm. MiRNA reverse transcription was conducted using Multiscribe RTkit (Biosystems, Spain). Reverse transcription conditions were as followings: reacting for 10 min at 25°C, 30 min at 48°C, and a final step of 5 min at 95°C. The PCR reactions were at 95°C for 5 min, followed by 40 cycles of 95°C for 15 s, 60°C for 30 s, and 72°C for 30 s. The relative expression levels were analyzed by the 2^-△△Ct^ method and all experiments were repeated three times.

### Protein isolation and western blotting analysis

Experimental monolayers were rinsed three times gently with PBS, and total protein was then isolated by RIPA lysis buffer (Beyotime Biotechnology, China) fortified with protease inhibitors (Roche, Switzerland). The extracting solutions were centrifuged at 12,000 *g* at 4°C for 20 min. An equal amount of protein was quantified with BCA™ Protein Assay Kit (Invitrogen). Lysates could be segregated on SDS-PAGE and transferred to nitrocellulose membranes. Subsequently, the membranes were blocked with 5% defatted milk for 3 h at 37°C to block nonspecific binding. After blocking, specific antibodies such as anti-Bcl-2 (No. ab112, Beyotime), anti-Bax (No. ab026, Beyotime), anti-caspase-3 (No. ab32499, Abcam, USA), anti-cleaved-caspase-3 (No. ab2302, Abcam), anti-Beclin-1 (No. ab62557, Abcam), anti-p62 (No. ab56416, Abcam), anti-LC-3B (No. ab48394, Abcam), anti-PI3K (No. ab151549, Abcam), anti-p-PI3K (No. ab138364, Abcam), anti-AKT (No. 4685, Cell Signaling, USA), anti-mTOR (No. ab2732, Abcam), anti-p-mTOR (No. sc-293132, Santa Cruz Biotechnology, USA), and anti-p-AKT (No. sc-271966, Santa Cruz Biotechnology) were added to the membranes. Different kinds of primary antibodies were incubated with the membranes separately at 4°C overnight. Tris buffered saline Tween (TBST) (Solarbio) was used to wash the membranes gently, which were then incubated with appropriate horseradish peroxidase-conjugated secondary antibodies for 1 h at room temperature. Finally, each protein was detected by Bio-Rad ChemiDoc™ XRS system (Bio-Rad), and the area of each band was quantified using Image Lab™ Software (Bio-Rad). β-actin (No. SAB5500001, Sigma, USA) was used as an endogenous protein for normalization. Each test was performed in triplicate.

### Statistical analysis

All experiments were repeated at least three times. The data are reported as means±SD and were analyzed using SPSS 19.0 statistical software (SPSS, USA). Statistical analyses were performed by one-way analysis of variance (ANOVA) or Student's *t*-test. A P value of <0.05 was considered statistically significant.

## Results

### Hypoxic injury was induced in H9c2 cells

To investigate the effect of hypoxia, H9c2 cells were treated in hypoxia for 0, 2, 4, 8, 16, and 24 h. As shown in Figure 1A, hypoxia had a time-dependent growth inhibition effect on H9c2 cells. Cell viability was down to 46.36% under hypoxia for 16 h (P<0.0001). Thus, hypoxia treatment of the following experiments was carried out for 16 h. Hypoxia significantly enhanced apoptosis of H9c2 cells from 2.86 to 14.84% (P=0003, Figure 1B). Hypoxia significantly increased the expression of Bax (P<0.0001) and cleaved-caspase-3 (P<0.0001), and decreased the expression of Bcl-2 (P=0.0013, Figure 1C and D). Meanwhile, the expression of Beclin-1 was increased (P=0.0002), the expression of p62 was decreased (P=0.0002), and the expression of LC-3 II/LC-3 I was increased (P=0.0001, Figure 1E and F). These results implied that hypoxia could induce apoptosis and autophagy in H9c2 cells.

**Figure 1.** Hypoxia (HYPO) triggered damage of H9c2 cells. **A**, Cell viability was detected by CCK-8 assay. **B**, Cell apoptosis was assessed by flow cytometry. **C** and **D**, Protein expression levels of Bcl-2, Bax, pro-caspase-3, cleaved-caspase-3, and β-actin, and (**E** and **F**) of Beclin-1, p62, LC-3-II, LC-I, and β-actin were measured by western blot assay. Data are reported as mean±SD (ANOVA or Student's *t*-test).

### PD reduced hypoxic injury of H9c2 cells

According to the results of CCK-8 assay, PD showed no toxic effect on H9c2 cells at the concentration of 10 μM, and cell viability was decreased at the concentrations of 15 (P=0.0001) and 20 μM (P=0.0007). On the other hand, PD increased cell viability in a dose-dependent manner under the treatment of hypoxia. Thus, optimal concentration of PD was 10 μM (Figure 2A). As shown in Figure 2B, PD increased cell viability in H9c2 cells stimulated by hypoxia in a dose-dependent manner. In addition, apoptosis rate of the PD-treated group decreased significantly compared with the hypoxia (HYPO) group (P=0.0009, Figure 2C). PD promoted the expression of Bcl-2 (P=0.0015), and decreased the expression of cleaved-caspase-3 (P=0.0038) and Bax (P=0.0019, Figure 2D and E). Furthermore, PD reduced the expression of Beclin-1 (P=0.0017) and the rate of LC-3 II/LC-3 I (P=0.0017). PD slightly increased the expression of p62 (P=0.0008) and showed no significant difference compared with the HYPO group (Figure 2F and G). These results demonstrated the PD could reduce the effect of hypoxia on H9c2 cells.

**Figure 2.** Polydatin (PD) reduced hypoxic injury of H9c2 cells. **A**, H9c2 cells were treated with PD at the concentrations of 1, 3, 10, 15, and 20 μM. **B**, H9c2 cells were pretreated by PD before hypoxia (HYPO). Cell viability was detected by CCK-8 assay. **C**, Cell apoptosis was assessed by flow cytometry. **D** and **E**, Western blot was used to measure the expression levels of Bcl-2, Bax, pro-caspase-3, and cleaved-caspase-3. **F** and **G**, Western blot was used to determine the expression levels of Beclin-1, p62, LC-3-II, and LC-I. Data are reported as mean±SD (ANOVA or Student's *t*-test).

### PD up-regulated the expression level of DGCR5

To investigate the relationship between PD and DGCR5 expression, H9c2 cells were treated by hypoxia alone or in combination with PD. The data suggested that the expression level of DGCR5 was proportional to the concentration of PD (P=0.0006 or P<0.0001, Figure 3). PD could up-regulate the expression level of DGCR5.

**Figure 3.** Polydatin (PD) increased the expression of DiGerorge syndrome critical region gene 5 (DGCR5) in hypoxia-induced (HYPO) injury of H9c2 cells measured by western blot. Data are reported as mean±SD (ANOVA or Student's *t*-test).

### PD reduced hypoxia-induced injury of H9c2 cells by means of up-regulation of DGCR5

In order to investigate the biological role of DGCR5, si-NC or si-DGCR5 was transfected into cells. Real-time quantitative PCR was utilized to reveal the transfection efficiency. The expression of DGCR5 was notably decreased by si-DGCR5 compared to si-NC (P<0.0001, Figure 4A). As shown in Figure 4B, PD significantly attenuated hypoxia-induced viability in the HYPO+PD+si-DGCR5 group compared to the HYPO+PD+si-NC group (P=0.0086). In addition, cell apoptosis was notably increased in the HYPO+PD+si-DGCR5 group compared to the HYPO+PD+si-NC group (P=0.0070, Figure 4C). The expressions of Bax (P=0.0066) and cleaved-caspase-3 were increased (P=0.0010), and the expression of Bcl-2 was decreased in the HYPO+PD+si-DGCR5 group compared to the HYPO+PD+si-NC group (P=0.0004, Figure 4D and E). These results indicated that PD reduced hypoxia-induced apoptosis in H9c2 cells by up-regulating the expression of DGCR5. In addition, the expression of Beclin-1 was increased (P=0.0037), the expression of p62 was decreased (P=0.0018), and the expression of LC-3 II/LC-3 I was highly increased in the HYPO+PD+si-DGCR5 group compared to the HYPO+PD+si-NC group (P=0.0009, Figure 4F and G). These results suggested PD inhibited the hypoxia-induced autophagy by up-regulating the expression of DGCR5.

**Figure 4.** Polydatin (PD) reduced hypoxia-induced (HYPO) injury by up-regulating the expression of DGCR5. **A**, The expression level of DGCR5 was detected by qRT-PCR. **B**, Cell viability was measured by CCK-8 assay. **C**, Apoptosis of H9c2 cells was measured by flow cytometry. **D** and **E**, Western blot analysis was used to measure the expression levels of Bcl-2, Bax, and cleaved-caspase-3. **F** and **G**, Western blot analysis was used to determine the expression levels of Beclin-1, p62, LC3-II, and LC3-I. Data are reported as mean±SD (ANOVA or Student's *t*-test).

### DGCR5 exerted its function though PI3K/AKT/mTOR and MEK/ERK signaling pathways in H9c2 cells

Western blot assay was done to analyze the total protein and phosphorylated protein expressions of PI3K, AKT, m-TOR, MEK, and ERK. As shown in Figure 5A and B, the rates of p/t-PI3K (P=0.0009), p/t-AKT (P=0.0029), and p/t-mTOR (P<0.0001) were inhibited in the HYPO group. Moreover, the rates were all higher in the HYPO+PD group compared to the HYPO group (P=0.0006, P=0.0002, or P<0.0001). In addition, the rates were decreased in the HYPD+PD+si-DGCR5 group compared to the HYPO+PD+si-NC group (P=0.0007, P=0.0022, or P<0.0001). Similarly, the rates of p/t-MEK and p/t-ERK were decreased in the HYPO group (P=0.0012 or P<0.0001), and the rates were reversed in the HYPO+PD group compared to the HYPO group (P<0.0001 or P=0.0002). Finally, the rates were attenuated in the HYPO+PD+si-DGCR5 group compared to the HYPO+PD+si-NC group (P=0.0021 or P<0.0001, Figure 5C and D). These results indicated that the effect of PD on the signaling pathways was eliminated by DGCR5 silencing.

**Figure 5.** Polydatin (PD) activated the PI3K/AKT/mTOR and MEK/ERK pathways. **A** and **B**, The total protein expression levels of PI3K, AKT, mTOR as well as phosphorylated PI3K, AKT, mTOR were analyzed by western blot. **C** and **D**, The total protein expression levels of MEK and ERK, as well as phosphorylated MEK and ERK were analyzed by western blot. Data are reported as mean±SD (ANOVA).

## Discussion

MI remains a primary health care problem worldwide (6) and is one of the most common causes of chronic heart failure (18). Previous research demonstrated that pretreatment with PD alleviated cardiac dysfunction *in vivo* (6). In this study, we cultured H9c2 cells with hypoxia to stimulate hypoxic damage *in vitro*. Furthermore, we provided evidence that PD could alleviate hypoxia-induced injury in H9c2 cells. PD decreased cell apoptosis and autophagy induced by hypoxia treatment in cardiomyocytes. Additionally, PD mobilized PI3K/AKT/mTOR and ERK/MEK signaling pathways by up-regulating the expression of DGCR5.

As a protective active substance, PD has shown target-specific molecular alterations in various cancers and has demonstrated encouraging results in treating MI (19). It has been reported that PD inhibited proliferation, invasion, and migration of laryngeal cancer, lung cancer, and hepatocellular carcinoma (20 [Bibr B21]–22). Furthermore, several studies demonstrated the function and mechanism of PD on MI. Zhang et al. (6) reported that PD protected cardiomyocytes from myocardial infarction injury by activating Sirt3.

Previous studies investigated the mechanism of PD and lncRNAs in diseases. For instance, Hu et al. reported that PD inhibited proliferation and apoptosis of doxorubicin-resistant osteosarcoma through lncRNA TUG1-mediated AKT pathway (19). Moreover, PD protected brain microvascular integrity and ameliorated stroke through the C/EBPβ/MALAT1/CREB/PGC-1α/PPARγ pathway via regulating MALAT1 (23). Thus, we hypothesized PD could play a role in MI by regulating lncRNA.

Autophagy is critical for accelerating protein turnover during cardiac remodeling and essential for preventing the accumulation of paraproteins or damaged organelles. Autophagy degenerates damaged protein aggregates and organelles, maintaining organelle function and protein quality. Low levels of moderated autophagy are vital for maintaining cellular function. Under the treatment of hypoxia, autophagy is acutely activated. Nonetheless, excessive autophagy is harmful to cells. Excessive autophagy leads to massive cell death ultimately leading to impaired function *in vivo* (24). We observed autophagy in H9c2 cells under the treatment of hypoxia as well as with pretreatment with PD. The data showed that PD raised the expression of Beclin-1 and the rate of LC-3 II/LC-3, and decreased the accumulation of p62. Previous reports showed that Beclin-1, p62, LC-3 II, and LC-3 I were autophagy-specific proteins (25), and the transformation of LC-3 I to LC-3 II is a distinct symbol of autophagic activity (26,27). Therefore, pretreatment with PD reduced autophagy induced by hypoxia in H9c2 cells.

The characteristics of cell apoptosis are cell contraction, cytoplasmic vesication, chromatin condensation, and DNA fragmentation, finally leading to cell destruction (28). Apoptosis usually depends on the expression of pro-apoptosis genes and anti-apoptosis genes (29). Many genes and proteins are related to the regulation of apoptosis such as Bax, Bak, wild-type p53, Bcl-2, Bcl-xl, and mutant p53 (30 [Bibr B31]–32). In a previous study, PD has been proven to prevent apoptosis in human umbilical vein endothelial cells (33). According to our research, PD prevented apoptosis in hypoxia-induced H9c2 cells. These results indicated that PD might reduce apoptosis and autophagy when it is used clinically to prevent MI.

Several lncRNAs have been reported to protect H9c2 cells against hypoxia-induced injury (34). DGCR5 is implicated in some other diseases. For instance, Liu et al. (35) reported the effect of DGCR5 on apoptosis and cell viability of cervical cancer. DGCR5 facilitated apoptosis in gastric cancer cells *in vitro* according to Xu et al. (16). Dong et al. (36) suggested that DGCR5 played an anti-apoptosis role in lung adenocarcinoma. Nevertheless, the function of DGCR5 in cardiomyocytes is not clear. In this study, we found that DGCR5 silence decreased cell viability and increased apoptosis. Furthermore, DGCR5 acted as a regulatory effector of PD, and PD inhibited hypoxia-induced injury via up-regulating the expression of DGCR5.

PI3K/AKT/mTOR is an acknowledged signaling pathway that regulates various biological functions in cardiomyocytes, such as cell viability, apoptosis, and autophagy of mammalian cells (24,37). Previous study pointed out that overexpression of Sox8 could activate the PI3K/AKT/mTOR signaling pathway in H9c2 cells and reduce hypoxia-induced injury (34). The present data suggested that DGCR5 activation of PI3K/AKT/mTOR pathway was necessary for PD-mediated inhibition of H9c2 cells apoptosis. PD induces the expression of DGCR5 to activate PI3K/AKT/mTOR signaling pathway.

MEK/ERK signaling pathway has been proven to participate in the regulation of cell autophagy (38) and cytoprotection (39). Wu et al. (40) suggested that cucurbitacin-induced hypertrophy was through activation of autophagy via MER/ERK1/2 signaling pathway in H9c2 cells. Our results indicated that PD induced autophagy and apoptosis in cardiomyocytes through the activation of the MEK/ERK signaling pathway. Furthermore, we proved the relationship between DGCR5 and MER/ERK signaling pathway, as DGCR5 up-regulated the expression of MEK and ERK.

In summary, our research showed that PD protected H9c2 cells from apoptosis and autophagy promoted by hypoxia. Moreover, we provided the evidence that PD protected cardiomyocytes via up-regulating the expression of DGCR5. In addition, the expression of DGCR5 activated PI3K/AKT/mTOR and MEK/ERK signaling pathways. Further *in vivo* experiments need to be conducted to prove the effect of PD. The molecular mechanism of PD and DGCR5 in myocarditis will be verified in a 3D *in vitro* model in the future. This study provided a novel strategy for clinical therapy of MI.
